# PSSPNN: PatchShuffle Stochastic Pooling Neural Network for an Explainable Diagnosis of COVID-19 with Multiple-Way Data Augmentation

**DOI:** 10.1155/2021/6633755

**Published:** 2021-03-08

**Authors:** Shui-Hua Wang, Yin Zhang, Xiaochun Cheng, Xin Zhang, Yu-Dong Zhang

**Affiliations:** ^1^School of Computer Science, Henan Polytechnic University, China, Henan 454001, China; ^2^School of Architecture Building and Civil Engineering, Loughborough University, Loughborough LE11 3TU, UK; ^3^School of Information and Communication Engineering, University of Electronic Science and Technology of China, Chengdu 611731, China; ^4^School of Science & Technology, Middlesex University, London NW4 4BT, UK; ^5^Department of Medical Imaging, The Fourth People's Hospital of Huai'an, Huai'an, Jiangsu Province 223002, China; ^6^School of Informatics, University of Leicester, Leicester LE1 7RH, UK

## Abstract

**Aim:**

COVID-19 has caused large death tolls all over the world. Accurate diagnosis is of significant importance for early treatment.

**Methods:**

In this study, we proposed a novel PSSPNN model for classification between COVID-19, secondary pulmonary tuberculosis, community-captured pneumonia, and healthy subjects. PSSPNN entails five improvements: we first proposed the n-conv stochastic pooling module. Second, a novel stochastic pooling neural network was proposed. Third, PatchShuffle was introduced as a regularization term. Fourth, an improved multiple-way data augmentation was used. Fifth, Grad-CAM was utilized to interpret our AI model.

**Results:**

The 10 runs with random seed on the test set showed our algorithm achieved a microaveraged F1 score of 95.79%. Moreover, our method is better than nine state-of-the-art approaches.

**Conclusion:**

This proposed PSSPNN will help assist radiologists to make diagnosis more quickly and accurately on COVID-19 cases.

## 1. Introduction

COVID-19 is a type of disease caused by a new strain of coronavirus. “CO” means corona, “VI” virus, and “D” disease. Up to 22 December 2020, COVID-19 has caused more than 78.0 million confirmed cases and over 1.71 million deaths (US 326.5 k, Brazil 188.2 k, India 146.1 k, Mexico 119.4 k, Italy 69.8 k, and UK 68.3 k).

To diagnose COVID-19, two methods exist: (i) real-time reverse transcriptase PCR with nasopharyngeal swab samples to test the existence of RNA fragments and (ii) chest imaging (CI) examines the evidence of COVID-19. The first type of rRT-PCR method needs to wait for a few days to get the results, while the second type of CI approach could get quick results within minutes. The CI approaches have several advantages compared to rRT-PCR. First, the swab may be contaminated [1, 2]. Second, CI can detect the lesions of lungs where “ground-glass opacity (GGO)” will be observed to distinguish COVID-19 from healthy subjects. Third, CI can provide an immediate result as soon as imaging is complete. Fourth, reports show that chest computed tomography (CCT), one type of CI approach, can detect 97% of COVID-19 infections [3].

Currently, there are three types of CI approaches: chest X-ray (CXR) [4], chest CT (CCT), and chest ultrasound (CUS) [5]. Among all three types of approaches, CCT can provide the finest resolution than the other two CI approaches, allowing visualization of extremely small nodules in the lung. The additional advantage of CCT is that it can provide high-quality, three-dimensional chest data where radiologists can clearly view the COVID-19 lesions, which may be obscure in the other two CI approaches.

However, manual labeling by human experts is tedious, labor-intensive, and time-consuming [6]. Besides, the labeling performances are easily affected by interexpert and intraexpert factors (e.g., emotion, tiredness, and lethargy). Moreover, the labeling throughputs of radiologists are not comparable with artificial intelligence (AI) models. For example, senior radiologists may diagnose one scanning within five minutes, but AI can analyze thousands of samples within one minute. Particularly, early lesions are small and similar to surrounding normal tissues, which make them more challenging to measure and hence can potentially be neglected by radiologists.

Traditional AI methods have successfully been applied in many medical fields. For instance, Wang et al. [7] chose wavelet packet Tsallis entropy as a feature descriptor and employed a real-coded biogeography-based optimization (RCBO) classifier. Jiang and Zhang [8] proposed a 6-level convolutional neural network (6L-CNN) for therapy and rehabilitation. Their performances were improved by replacing the traditional rectified linear unit with a leaky rectified linear unit. Fulton et al. [9] used ResNet-50 (RN-50) to classify Alzheimer's disease with and without imagery. The authors found that ResNet-50 models help identify AD patients. Guo and Du [10] utilized a ResNet-18 (RN-18) model to recognize thyroid ultrasound standard plane (TUSP), achieving a classification accuracy of 83.88%. The experiments verified the effectiveness of RN-18. The aforementioned four algorithms can be transferred to the multiclass classification task of COVID-19 diagnosis.

On the COVID-19 datasets, several recent publications reported promising results. For example, Cohen et al. [11] proposed a COVID severity score network (CSSNet), which achieved a mean absolute error (MAE) of 1.14 on geographic extent score and an MAE of 0.78 on lung opacity score. Li et al. [12] developed a fully automatic model (COVNet) to detect COVID-19 using chest CT and evaluated its performance. Wang et al. [13] proposed a 3D deep convolutional neural network to detect COVID-19 (DeCovNet). Zhang et al. [14] proposed a seven-layer convolutional neural network for COVID-19 diagnosis (7L-CCD). Their performance achieved an accuracy of 94.03 ± 0.80 for the binary classification task (COVID-19 against healthy subjects). Ko et al. [15] proposed a fast-track COVID-19 classification network (FCONet). For the sake of the page limit, the details of those methods are not described, but we shall compare our method with those state-of-the-art methods in the following sections. Wang et al. [16] presented a CCSHNet via transfer learning and discriminant correlation analysis.

Our study's inspiration is to improve recognition performances of COVID-19 infection in CCT images by developing a novel deep neural network, PSSPNN, short for PatchShuffle stochastic pooling neural network. Our contributions entail the following five angles:

- The “*n*-conv stochastic pooling module (NCSPM)” is proposed, which comprises *n*-times repetitions of convolution layers and batch normalization layers, followed by stochastic pooling
- A novel “stochastic pooling neural network (SPNN)” is proposed, the structure of which is inspired by VGG-16
- A more advanced neural network, PatchShuffle SPNN (PSSPNN), is proposed where PatchShuffle is introduced as the regularization term in the loss function of SPNN
- An improved multiple-way data augmentation is utilized to help the network avoid overfitting
- Grad-CAM is used to show the explainable heatmap, which displays association with lung lesions

## 2. Dataset

This retrospective study was exempt by Institutional Review Board of local hospitals. Four types of CCT were used: (i) COVID-19-positive patients, (ii) community-acquired pneumonia (CAP), (iii) second pulmonary tuberculosis (SPT), and (iv) healthy control (HC). Three diseased classes (COVID-19, CAP, and SPT) were chosen since they are all infectious diseases of the chest regions. We intend to include the fifth category (chest tumors) in our future studies.

For each subject, *n*(*k*) slices of CCT were chosen via a slice level selection (SLS) method. For the three diseased groups (COVID-19, CAP, and SPT represented as *k* = {1, 2, 3}), the slice displaying the largest number of lesions and size was chosen. For HC subjects (*k* = 4), any slice within the 3D image was randomly chosen. The slice-to-subject ratio $\bar{n}$ is defined as

(1) $$\begin{array}{c} \bar{n}\left(k\right)=\frac{N_{S}\left(k\right)}{N_{P}\left(k\right)},k=1,\cdots ,4, \end{array}$$

where *N*_*S*_ stands for the number of slices via the SLS method and *N*_*P*_ is the number of patients.

In all, we enrolled 521 subjects and produced 1164 slice images using the SLS method.  Table 1 lists the demographics of the four-category subject cohort with the values of triplets $\left[\bar{n},N_{P},N_{S}\right]$, where $\bar{n}$ of the total set equals to 2.23.

Three experienced radiologists (two juniors: *𝒞*_1_ and *𝒞*_2_ and one senior: *𝒞*_3_) were convened to curate all the images. Suppose *x*^CCT^ means one CCT scan, *Y* stands for the labeling of each individual radiologist. The last labeling *Y*^*F*^ of the CCT scan *x*^CCT^ is obtained by

(2) $$\begin{array}{c} Y^{F}\left[x^{\text{CCT}}\right]=\left\{\begin{array}{cc} Y\left[C_{1},x^{\text{CCT}}\right] & Y\left[C_{1},x^{\text{CCT}}\right]==Y\left[C_{2},x^{\text{CCT}}\right]\\ \text{MAV}\left\{Y^{\text{all}}\left[x^{\text{CCT}}\right]\right\} & \text{otherwise} \end{array}\right., \end{array}$$

where MAV denotes majority voting and *Y*^all^ the labeling of all radiologists, *viz.*,

(3) $$\begin{array}{c} Y^{\text{all}}\left[x^{\text{CCT}}\right]=\left[Y\left(C_{1},x^{\text{CCT}}\right),Y\left(C_{2},x^{\text{CCT}}\right),Y\left(C_{3},x^{\text{CCT}}\right)\right]. \end{array}$$

The above two equations mean that in situations of disagreement between the analyses of two junior radiologists (*𝒞*_1_, *𝒞*_2_), we consult a senior radiologist (*𝒞*_3_) to reach a MAV-type consensus. Data is available on request due to privacy/ethical restrictions.

## 3. Methodology

Table 2 gives the abbreviation and full meanings in this study.  Section 3.1 shows the preprocessing procedure. Sections 3.2–3.5 offer four improvements. Finally, Section 3.6 gives the implementation, measure indicators, and explainable technology used in our method.

### 3.1. Preprocessing

The original raw dataset contained |*V*| slice images {*v*_*a*_(*i*), *i* = 1, 2, ⋯, |*V*|}. The size of each image was size[*v*_*a*_(*i*)] = 1024 × 1024 × 3.  Figure 1 presents the pipeline for preprocessing of this dataset.

First, the color CCT images of four classes were converted into grayscale by retaining the luminance channel and obtaining the grayscale data set *V*_*B*_:

(4) $$\begin{array}{c} V_{B}=O_{\text{gray}}\left(V_{A}\right)=\left\{v_{b}\left(1\right),v_{b}\left(2\right),\cdots ,v_{b}\left(i\right),\cdots v_{b}\left(\left|V\right|\right)\right\}, \end{array}$$

where *O*_gray_ means the grayscale operation.

In the second step, the histogram stretching (HS) was utilized to increase the contrast of all images. Take the *i*-th image *v*_*b*_(*i*), *i* = 1, 2, ⋯, |*V*| as an example; its minimum and maximum grayscale values *v*_*b*_^*l*^(*i*) and *v*_*b*_^*h*^(*i*) were calculated as follows:

(5) $$\begin{array}{c} \left\{\begin{array}{c} v_{b}^{l}\left(i\right)=\min_{w=1}^{W_{B}}\min_{h=1}^{H_{B}}\min_{c=1}^{C_{B}}v_{b}\left(i\;|\;w,h,c\right),\\ v_{b}^{h}\left(i\right)=\max_{w=1}^{W_{B}}\max_{h=1}^{H_{B}}\max_{c=1}^{C_{B}}v_{b}\left(i\;|\;w,h,c\right). \end{array}\right. \end{array}$$

Here, (*w*, *h, c*) means the index of width, height, and channel directions along image *v*_*b*_(*i*), respectively. (*W*_*B*_, *H*_*B*_, *C*_*B*_) means the maximum values of width, height, and channel to the image set *V*_*B*_. The new histogram stretched image set *V*_*C*_ was calculated as follows:

(6) $$\begin{array}{c} V_{C}=O_{\text{HS}}\left(V_{B}\right)=\left\{v_{c}\left(i\right)≝\frac{v_{b}\left(i\right)-v_{b}^{l}\left(i\right)}{v_{b}^{h}\left(i\right)-v_{b}^{l}\left(i\right)}\right\}, \end{array}$$

where *O*_HS_ stands for the HS operation.

In the third step, cropping was performed to remove the checkup bed at the bottom area and eliminate the texts at the margin regions. Cropped dataset *V*_*D*_ is yielded as

(7) $$\begin{array}{c} V_{D}=O_{\text{crop}}\left(V_{C},\left[a_{1},a_{2},a_{3},a_{4}\right]\right)=\left\{v_{d}\left(1\right),v_{d}\left(2\right),\cdots ,v_{d}\left(i\right),\cdots ,v_{d}\left(\left|V\right|\right)\right\}, \end{array}$$

where *O*_crop_ represents crop operation. Parameters (*a*_1_, *a*_2_, *a*_3_, *a*_4_) mean pixels to be cropped from four directions of the top, bottom, left, and right, respectively (unit: pixel).

In the fourth step, each image was downsampled to a size of [*W*_*E*_, *H*_*E*_], obtaining the resized image set *V*_*E*_ as

(8) $$\begin{array}{c} V_{E}=O_{\text{DS}}\left(V_{D},\left[W_{E},H_{E}\right]\right)=\left\{v_{e}\left(1\right),v_{e}\left(2\right),\cdots ,v_{e}\left(i\right),\cdots v_{e}\left(\left|V\right|\right)\right\} \end{array}$$

where *O*_DS_ : *a* ↦ *b* represents the downsampling (DS) procedure, in which *b* stands for the downsampled image of the raw image *a*.

Figure 2 displays example images of the four categories, in which three are diseased, and one is healthy. The original size of each image in *V*_*A*_ is 1024 × 1024 × 3, and the final preprocessed image is 256 × 256 × 1.

### 3.2. Improvement I: *n*-conv Stochastic Pooling Module

First, stochastic pooling (SP) [17] was introduced. In the standard convolutional neural networks, pooling is an essential component after each convolution layer, which was applied to reduce the size of feature maps (FMs). SP was shown to give better performance than average pooling and max pooling in recent publications [18–21]. Recently, strided convolution (SC) is commonly used, which also can shrink the FMs [22, 23]. Nevertheless, SC could be considered a simple pooling method, which always outputs the region's fixed-position value [24].

Suppose we have a postconvolution FM *𝔽* = *f*_*ij*_(*i* = 1, ⋯, *M* × *P*, *j* = 1, ⋯, *N* × *Q*). The FM can be separated into *M* × *N* blocks, in which every block has the size of *P* × *Q*. Now we focus on the block *B*_*mn*_ = {*b*(*x*, *y*), *x* = 1, ⋯, *P*, *y* = 1, ⋯, *Q*} which stands for the *m*-th row and *n*-th column blocks.

The strided convolution (SC) traverses the input activation map with the strides, which equals the size of the block (*P*, *Q*), so here its output is set to

(9) $$\begin{array}{c} B_{mn}^{\text{SC}}=b\left(1,1\right). \end{array}$$

The l2-norm pooling (L2P), average pooling (AP), and max pooling (MP) generate the l2-norm value, average value, and maximum value within the block *B*_*mn*_, respectively.

(10) $$\begin{array}{c} \left\{\begin{array}{c} B_{mn}^{\text{L}2\text{P}}=\sqrt{\frac{\sum_{x=1}^{P}\sum_{y=1}^{Q}b^{2}\left(x,y\right)\;}{P\times Q}},\\ B_{mn}^{\text{AP}}=\frac{1}{P\times Q}\overset{P}{\underset{x=1}{\sum }}\overset{Q}{\underset{y=1}{\sum }}b\left(x,y\right),\\ B_{mn}^{\text{MP}}=\max_{x=1}^{P}\max_{y=1}^{Q}b\left(x,y\right). \end{array}\right. \end{array}$$

The SP provides a solution to the shortcomings of AP and MP. The AP outputs the average, so it will downscale the largest value, where the important features may sit on. On the other hand, MP reserves the maximum value but worsens the overfitting problem. SP is a three-step procedure. First, it generates the probability map (PM) for each entry in the block *B*_*mn*_.

(11) $$\begin{array}{c} \left\{\begin{array}{c} p_{m}\left(x,y\right)=\frac{b\left(x,y\right)}{\sum_{x=1}^{P}\sum_{y=1}^{Q}b\left(x,y\right)},\\ s.t.\overset{P}{\underset{x=1}{\sum }}\overset{Q}{\underset{y=1}{\sum }}p_{m}\left(x,y\right)=1, \end{array}\right. \end{array}$$

where *p*_*m*_(*x*, *y*) stands for the PM value at pixel (*x*, *y*).

In the second step, create a random variable *r* that takes the discrete probability distribution (DPD) as

(12) $$\begin{array}{c} \left\{\begin{array}{c} \mathrm{Pr}\left[r=\left(1,1\right)\right]=p_{m}\left(1,1\right)\;\mathrm{Pr}\left[r=\left(1,2\right)\right]=p_{m}\left(1,2\right)\;\cdots \;\mathrm{Pr}\left[r=\left(1,Q\right)\right]=p_{m}\left(1,Q\right),\\ \mathrm{Pr}\left[r=\left(2,1\right)\right]=p_{m}\left(2,1\right)\;\mathrm{Pr}\left[r=\left(2,2\right)\right]=p_{m}\left(2,2\right)\;\cdots \;\mathrm{Pr}\left[r=\left(2,Q\right)\right]=p_{m}\left(2,Q\right),\\ \cdots \;\cdots \;\cdots \;\cdots \\ \mathrm{Pr}\left[r=\left(P,1\right)\right]=p_{m}\left(P,1\right)\;\mathrm{Pr}\left[r=\left(P,2\right)\right]=p_{m}\left(P,2\right)\;\cdots \;\mathrm{Pr}\left[r=\left(P,Q\right)\right]=p_{m}\left(P,Q\right), \end{array}\right. \end{array}$$

where Pr represents the probability.

In the third step, a sample *r*_0_ is drawn from the random variable *r*, and the corresponding position pos(*r*_0_) = (*x*_*r*_0__, *y*_*r*_0__). Then, the output of SP is at location pos(*r*_0_), namely,

(13) $$\begin{array}{c} B_{mn}^{\text{SP}}=b\left(x_{r_{0}},y_{r_{0}}\right). \end{array}$$

Figure 3 presents the comparison of four different pooling techniques. The top left shows the raw FM in which the pooling will take place at a 3 × 3 kernel. If we take the top-right block (in an orange rectangle) as an example, the L2P outputs 4.96, while AP and MP output 4.08 and 9.3, respectively. For the SP method, it will first generate the PM and then sample a position based on the PM (see the red fonts), and thus, SP outputs the value of 6.

A new “n-conv stochastic pooling module” (NCSPM) is proposed in this study based on the SP layer discussed in previous paragraphs. The NCSPM entails *n*-repetitions of a conv layer and a batch normalization layer, followed by an SP layer.  Figure 4 shows the schematic of the proposed NCSPM module. In this study, *n* = 1∨2, since we experimented using *n* = 3, but the performance using *n* = 3 did not improve.

### 3.3. Improvement II: Stochastic Pooling Neural Network

The second improvement of this study is to propose a stochastic pooling neural network (SPNN), whose structure was inspired by VGG-16 [25]. In VGG-16, the network used small kernels instead of large kernels and always used 2 × 2 filters with a stride of 2 for pooling. In the end, VGG-16 has two fully connected layers (FCLs).

This proposed SPNN will follow the same structure design of VGG-16 but using the NCSPM module to replace the convolution block in VGG-16. The details of SPNN are shown in Table 3, where NWL means the number of weighted layers, HS is the hyperparameter size, and FMS is the feature map size.

Compared to ordinary CNN, the advantages of SPNN are two folds: (i) SPNN helps prevent overfitting; (ii) SPNN is parameter-free. (iii) SPNN can be easily combined with other advanced techniques, such as batch normalization and dropout. In total, we create this 11-layer SPNN. We have attempted to insert more NCSPMs or more FCLs, which does not show performance improvement but more computation burden. The structure of the proposed model is summarized in Table 3. The [*c*_1_ × *c*_1_, *c*_2_] × *c*_3_ related to NCSPM stands for *c*_3_ repetitions of *c*_2_ filters with size of *c*_1_ × *c*_1_. For the FCL, the *c*_1_ × *c*_2_, *c*_3_ × *c*_4_ stands for a weight matrix is with size of *c*_1_ × *c*_2_ and a bias matrix is with size of *c*_3_ × *c*_4_. In the last column of Table 3, the format of *c*_1_ × *c*_2_ × *c*_3_ represents the feature map's size in three dimensions: height, width, and channel. Directly using transfer learning is another alternative.

In this study, we chose to create a custom neural network by designing its structure and training the whole network using our own data. The reason is some reports have shown this “built your own network from scratch” can achieve better performance than transfer learning [26, 27].

### 3.4. Improvement III: PatchShuffle SPNN

Kang et al. [28] presented a new PatchShuffle method. In each minibatch, images and feature maps undergo a transformation such that pixels with that patch are shuffled. By generating fake images/feature maps with interior order-less patches, PatchShuffle creates local variations and reduces the possibility of the AI model overfitting. Therefore, PatchShuffle is a beneficial supplement to various existing training regularization methods [28].

Assume there is a matrix *X* of *M* × *M* entries. A random variable *v* controls whether the matrix *X* to be PatchShuffled or not. The random variable *v* obeys the Bernoulli distribution

(14) $$\begin{array}{c} v\sim \text{Bernoulli}\left(\varepsilon \right). \end{array}$$

Namely, *v* = 1 with probability *ε*, and *v* = 0 with probability 1 − *ε*. The resulted matrix $\hat{X}$ is written as

(15) $$\begin{array}{c} \hat{X}=\left(1-v\right)X+vF^{\text{PS}}\left(X\right), \end{array}$$

where *F*^PS^ is the PatchShuffle operation. Suppose the size of each patch is *m* × *m*, we can express the matrix *X* as

(16) $$\begin{array}{c} X=\left[\begin{array}{cccc} x_{11} & x_{12} & \cdots & x_{1,M/m}\\ x_{21} & x_{22} & \cdots & x_{2,M/m}\\ \vdots & \vdots & \ddots & \vdots \\ x_{M/m,1} & x_{M/m,2} & \cdots & x_{M/m,M/m} \end{array}\right], \end{array}$$

where *x*_*ij*_ stands for a nonoverlapping patch at *i*-th row and *j*-th column. The PatchShuffle transformation works on every patch.

(17) $$\begin{array}{c} F^{\text{PS}}\left(X\right)=\left\{F^{\text{PS}}\left(x_{ij}\right),i=1,\cdots ,\frac{M}{m},j=1,\cdots ,\frac{M}{m}\right\}. \end{array}$$

The shuffled patch is formulated as

(18) $$\begin{array}{c} F^{\text{PS}}\left(x_{ij}\right)=e_{ij}\times x_{ij}\times e_{ij}^{\prime }, \end{array}$$

where *e*_*ij*_ is the row permutation matrix and *e*_*ij*_′ is the column permutation matrix [29]. In practice, a randomly shuffle operation is used to replace the row and column permutation operation. Each patch will undergo one of the *m*^2^! possible permutations.

We proposed integrating PatchShuffle into our SPNN, and this new network model is named as PatchShuffle stochastic pooling neural network (PSSPNN). The PatchShuffle operation acts on both the input image layer (see grayscale image Figure 5 and colorful image Figure 6 with different values of *m*) and the feature maps of all the convolutional layers (9 conv layers from NCSPM-1 to NCSPM-5).

The schematics of building PSSPNN from the SPNN are drawn in Figure 7, where either inputs or feature maps are randomly selected to undergo the PatchShuffle operation. To reach the best bias-variance trade-off, only a small percentage (*ε*) of the images/feature maps will undergo *F*^PS^ operation.

For simplicity, we consider the PatchShuffling images as an example, and the training loss function *ℓ* of the proposed PSSPNN is written as

(19) $$\begin{array}{c} \ell^{\text{PSSPNN}}\left(X,y,W\right)=\left(1-v\right)\ell \left(X,y,W\right)+v\ell \left[F^{\text{PS}}\left(X\right),y,W\right], \end{array}$$

where *ℓ* stands for the ordinary loss function and *ℓ*^PSSPNN^ the loss function of PSSPNN. **X** represents the original images and *F*^PS^(**X**) the PatchShuffled images. The label is symbolized as *y*, and the weights are symbolized as *𝒲*.

Considering the extreme situations when *v* = 0∨1, we have

(20) $$\begin{array}{c} \ell^{\text{PSSPNN}}\left(X,y,W\right)=\left\{\begin{array}{cc} \ell \left(X,y,W\right) & v=0,\\ \ell \left[F^{\text{PS}}\left(X\right),y,W\right] & v=1, \end{array}\right. \end{array}$$

which means the loss function degrades to ordinary loss function when *v* = 0, and meanwhile, the loss function equals to training all images PatchShuffled when *v* = 1. Taking mathematical expectation of *v*, equation (19) turns to

(21) $$\begin{array}{c} \frac{1}{1-\varepsilon }E_{v}\ell^{\text{PSSPNN}}\left(X,y,W\right)=\ell \left(X,y,W\right)+\frac{\varepsilon }{1-\varepsilon }\ell \left[F^{\text{PS}}\left(X\right),y,W\right], \end{array}$$

where *ε*/1 − *εℓ*[*F*^PS^(**X**), *y*, *𝒲*] acts as a regularization term.

### 3.5. Improvement IV: Improved Multiple-Way Data Augmentation

This small four-category dataset makes our AI model prone to overfitting. In order to alleviate the overfitting and handle the low sample-size problem, the multiple-way data augmentation (MDA) [30] method was chosen and further improved. In the original 14-way MDA [30], the authors used seven different data augmentation (DA) techniques to the raw image and its horizontal image. Their seven DA techniques are as follows: noise injection, horizontal shear, vertical shear, rotation, Gamma correction, scaling, and translation.

Figure 8 shows a 16-way data augmentation method. The difference between the proposed 16-way DA with the traditional 14-way DA is that we add the salt-and-pepper noise (SAPN). Although the SAPN defies intuition as it never takes place in realistic CCT images, we found that it can increase performance. The same observation was reported by Li et al. [31], where the authors used salt and pepper noise for the identification of early esophageal cancer.  Table 4 shows the pseudocode of this proposed 16-way improved data augmentation.

(22) $$\begin{array}{c} v\left(i\right)\mapsto D\left(i\right)=S\left\{\begin{array}{cc} v\left(i\right) & M\left[v\left(i\right)\right]\\ \underset{k=1,..,8}{S}\underset{W}{\underset{⏟}{f_{k}^{\text{DA}}\left[v\left(i\right)\right]}} & \underset{k=1,..,8}{S}\underset{W}{\underset{⏟}{f_{k}^{\text{DA}}\left\{M\left[v\left(i\right)\right]\right\}}} \end{array}\right\}, \end{array}$$

where *W* = 30 in this study. We tested a greater value of *W*, but it does not bring about significant improvement. Hence, one image *v*(*i*) will generate |*𝔻*(*i*)| = 16*W* + 2 = 482 images (including original image), as shown in Figure 8.

**Step 1 .**

Eight geometric or photometric DA transforms were utilized on raw image *v*(*i*), as shown in Figure 8. We use *f*_*k*_^DA^, *k* = 1, ⋯, 8 to denote each DA operation. Note each DA operation *f*_*k*_^DA^ will yield *W* new images. So, for a given image *v*(*i*), we will produce an enhanced dataset $\underset{k=1,..,8}{𝕊}f_{k}^{\text{DA}}\left[v\left(i\right)\right]$, where *𝕊* stands for concatenation function.

**Step 2 .**

Horizontal mirror image is generated as *M* [*v*(*i*)], where *M* means horizontal mirror function.

**Step 3 .**

The raw image *v*(*i*), the mirrored image *M* [*v*(*i*)], all the above 8-way DA results of raw image $\underset{k=1,..,8}{𝕊}f_{k}^{\text{DA}}\left[v\left(i\right)\right]$, and 8-way DA results of horizontal mirrored image $\underset{k=1,..,8}{𝕊}f_{k}^{\text{DA}}\left\{\text{M}\left[v\left(i\right)\right]\right\}$ are combined. Mathematically, one training image *v*(*i*) will generate to a dataset *𝔻*(*i*), which contains 16*W* + 1 new images.

Taking Figure 2(a) as an example raw image, Figure 9 shows the 8-way DA results, i.e., *f*_*k*_^DA^[*v*(*i*)], *k* = 1, ⋯, 8. Due to the page limit, the mirror image and its corresponding 8-way DA results are not shown here.

### 3.6. Implementation, Measure, and Explainability

Table 5 itemizes the nontest and test sets for each category. The whole dataset *V* contains four nonoverlapping categories *V* = {*V*_1_, *V*_2_, *V*_3_, *V*_4_}. For each category, the dataset will be split into nontest set and test set *V*_*k*_ → {*V*_*k*_^ntest^, *V*_*k*_^test^}, *k* = 1, 2, 3, 4.

(23) $$\begin{array}{c} V=\left[\begin{array}{c} V_{1}\\ V_{2}\\ V_{3}\\ V_{4} \end{array}\right]=\left[\begin{array}{cc} V^{\text{ntest}} & V^{\text{test}} \end{array}\right]=\left[\begin{array}{cc} V_{1}^{\text{ntest}} & V_{1}^{\text{test}}\\ V_{2}^{\text{ntest}} & V_{2}^{\text{test}}\\ V_{3}^{\text{ntest}} & V_{3}^{\text{test}}\\ V_{4}^{\text{ntest}} & V_{4}^{\text{test}} \end{array}\;\right]. \end{array}$$

Our experiment entails two phases. At phase I, 10-fold cross-validation was used for validation on the nontest set to select the best hyperparameters and best network structure. The 16-way DA was used on the training set of 10-fold cross-validation. The hyperparameter of the proposed PSSPNN was determined over the nontest set *V*^ntest^. Afterward at phase II, we train our model using the nontest set *V*^ntest^ 10 times with different initial seeds and attain the test results over the test set *V*^test^. After combining the *R*^test^ runs, we attain a summation of the test confusion matrix (TCM) *D*^test^. Table 5 shows the dataset splitting, where |*x*| stands for the number of elements in the dataset *x*.

The ideal TCM is a diagonal matrix with the form of

(24) $$\begin{array}{c} D_{\text{ideal}}^{\text{test}}=R^{\text{test}}\times \left[\begin{array}{cccc} \left|V_{1}^{\text{test}}\right| & 0 & 0 & 0\\ 0 & \left|V_{2}^{\text{test}}\right| & 0 & 0\\ 0 & 0 & \left|V_{3}^{\text{test}}\right| & 0\\ 0 & 0 & 0 & \left|V_{4}^{\text{test}}\right| \end{array}\right], \end{array}$$

in which all the off-diagonal elements are zero, meaning no prediction errors. In realistic scenarios, the AI model will make errors, and the performance is calculated per category. For each class *z* = 1, ⋯, 4, we set the label of that class as *positive*, and the labels of all the rest classes as *negative*. Three performance metrics (sensitivity, precision, and F1 score) per category are defined below:

(25) $$\begin{array}{c} \left\{\begin{array}{c} \text{Sen}\left(z\right)=\frac{\text{TP}\left(z\right)}{\text{TP}\left(z\right)+\text{FN}\left(z\right)},\\ \text{Prc}\left(z\right)=\frac{\text{TP}\left(z\right)}{\text{TP}\left(z\right)+\text{FP}\left(z\right)},\\ \text{F}1\left(z\right)=\frac{2*\text{Prc}\left(z\right)*\text{Sen}\left(z\right)}{\text{Prc}\left(z\right)+\text{Sen}\left(z\right)}. \end{array}\right. \end{array}$$

The performance can be measured over all four categories. The microaveraged (MA) F1 (symbolized as F1_*μ*_) is used since our dataset is slightly unbalanced:

(26) $$\begin{array}{c} \text{F}1_{\mu }=\frac{2*\mathrm{Pr}c_{\mu }*\text{Se}{\text{n}}_{\mu }}{\mathrm{Pr}c_{\mu }+\text{Se}{\text{n}}_{\mu }}, \end{array}$$

where

(27) $$\begin{array}{c} \left\{\begin{array}{c} \text{Se}{\text{n}}_{\mu }=\frac{\sum_{z=1}^{4}\text{T}\text{P}\left(z\right)}{\sum_{z=1}^{4}\text{T}\text{P}\left(z\right)+\text{FN}\left(z\right)},\\ \mathrm{Pr}c_{\mu }=\frac{\sum_{z=1}^{4}\text{T}\text{P}\left(z\right)}{\sum_{z=1}^{4}\text{T}\text{P}\left(z\right)+\text{FP}\left(z\right)}. \end{array}\right. \end{array}$$

Finally, gradient-weighted class activation mapping (Grad-CAM) [32] was employed to provide explanations on how our model makes the decision. It exploits the gradient of the categorization score regarding the convolutional features decided by the deep model to visualize the regions of the image that are the most vital for the image classification task [33]. The output of NCSPM-5 in Table 3 was used for Grad-CAM.

## 4. Experiments, Results, and Discussions

The experiment was carried out on the programming platform of Matlab 2020b. The programs ran on Windows 10 with 16GB RAM and 2.20GHz Intel Core i7-8750H CPU. The performances are reported over the test set with 10 runs.

### 4.1. Comparison of SPNN and Other Pooling Methods

In the first experiment, we compared the proposed SPNN with four standard CNNs with different pooling methods. The first CNN uses strided convolution in five modules to replace the stochastic pooling. The second to fourth comparison CNN models use L2P, AP, and MP, respectively. Those four baseline methods are called SC-CNN, L2P-CNN, AP-CNN, and MP-CNN, respectively. The results of 10 runs over the test set are shown in Table 6. The bar plot is displayed in Figure 10, where “*k*-*S*,” “*k*-*P*,” and “”*k*-F1” stand for the sensitivity, precision, and F1 score for category *k* ∈ {1, 2, 3, 4}.

The results in Table 6 and Figure 10 are coherent with our expectation that SPNN obtained the best results among all FM reduction approaches. The SPNN arrives at the sensitivities of all four categories are 98.07%, 91.79%, 94.92%, and 95.25%, respectively. The precisions of all four categories are 94.59%, 95.19%, 94.92%, and 95.40%, respectively. The F1-scores of the four categories are 96.30%, 93.45%, 94.92%, and 95.32%, respectively. The overall microaveraged F1 is 95.02%.

In terms of microaveraged F1, the second-best algorithm is MP-CNN, which obtains a microaveraged F1 score of 93.91%. The third best is AP-CNN, with a microaveraged F1 score of 93.18%. The two comparably worst algorithms are SC-CNN and L2P-CNN, with the microaveraged F1 scores of 92.40% and 92.53%, respectively.

SPNN obtains the best results because SP can prevent overfitting [17], which is the main shortcoming of max pooling. On the other hand, AP and L2P will average out the maximum activation values, which will impair the performances of convolutional neural network models. For SC-CNN, it only uses one quarter information of the input FM, and therefore may neglect those greatest values [34]. In all, this proposed SPNN can be regarded as an improved version of vanilla CNN models, where the SP is used to replace traditional MP.

### 4.2. PSSPNN versus SPNN

In this second experiment, we compared our two proposed network models, PSSPNN against SPNN, to validate the effectiveness of PatchShuffle. The results of 10 runs over the test set with different combinations of hyperparameters are shown in Table 7, and the 3D bar chart is shown in Figure 11. The optimal hyperparameter we found from the 10-fold cross-validation of the nontest set is *ε* = 0.05 and patch size is 2 × 2, which are coherent with reference [28].

In addition, the PSSPNN with optimal hyperparameter is compared with SPNN. The results are shown in Table 8. From the table, we can observe that PSSPNN provides better F1 values for all four categories and the overall microaverage, which shows the effectiveness of PatchShuffle. The reason is PatchShuffle adds regularization terms [28] in the loss function, and thus can improve the generalization ability of our SPNN model.

### 4.3. Comparison to State-of-the-Art Approaches

We compared our proposed PSSPNN method with 9 state-of-the-art methods: RCBO [7], 6L-CNN [8], RN-50 [9], RN-18 [10], CSSNet [11], COVNet [12], DeCovNet [13], 7L-CNN-CD [14], and FCONet [15]. All the comparison was carried on the same test set of 10 runs. The comparison results are shown in Table 9.

For ease of comparison, Figure 12 only compares the microaveraged F1 (MA F1) score of all algorithms, from which we can observe this proposed PSSPNN achieves the best performance among all the algorithms. This experiment is a simulation-based comparison. In the future, we will apply our algorithm to rigorous clinical testing and verification.

### 4.4. Explainability of Proposed PSSPNN

We take Figure 2 images as examples; the heatmaps of those four images are shown in Figures 13(a)–13(d), and the manual delineation, shown in Figures 13(e)–13(h), delineates the lesions of the three disease samples. Note there are no lesions of healthy control (HC) image. The NCSPM-5 feature map in PSSPNN was used to generate heatmaps with the Grad-CAM approach.

We can observe from Figure 13 that the heatmaps via our PSSPNN model and Grad-CAM can capture the lesions effectively and meanwhile neglect those nonlesion regions. Traditionally, AI is regarded as a “black box,” which impairs its widespread usage, e.g., the black box properties of traditional AI are problematic for the FDA. Nevertheless, with the help of explainability of modern AI techniques [35], the radiologist and patients will gain confidence in our proposed AI model, as the heatmap provides a clear and understandable interpretation of how AI predicts COVID-19 and other chest infectious disease from healthy subjects, which was also stated in reference [36]. Many new AI-based anatomic pathological systems now pass through FDA approval, such as whole slide images (WSI) [37], since the doctors know the relationships between the diagnosis and the explained answer.

In the future, the explainability of our proposed AI model can be used in patient monitoring [38] and health big data [39]. Some novel network improvement and signal processing techniques may help our AI model in future researches, such as filters [40, 41], fuzzy [42, 43], edge computing [44], knowledge-aid [45, 46], autofocus [47], graph integration, and cross-domain knowledge exploitation [48–50].

## 5. Conclusion

In this paper, we proposed a PSSPNN, which entails five improvements: (i) proposed NCSPM module, (ii) usage of stochastic pooling, (iii) usage of PatchShuffle, (iv) improved multiple-way data augmentation, and (v) explainability via Grad-CAM. Those five improvements enable our AI model to deliver improved performances compared to 9 state-of-the-art approaches. The 10 runs on the test set showed our algorithm achieved a microaveraged F1 score of 95.79%.

There are three shortcomings of our method, which will be resolved in the future: (i) the dataset currently contains three chest infectious diseases. In the future, we shall try to include more classes of chest diseases, such as thoracic cancer. (ii) Some new network techniques and models are not tested, such as transfer learning, wide network module design, attention mechanism, and graph neural network. Those advanced AI technologies will be studied. (iii) Our model does not go through strict clinical validation, so we will attempt to release our software to hospitals and get feedback from radiologists and consultants.

## Figures and Tables

**Figure 1:** Illustration of preprocessing.

**Figure 2:** Samples of four categories (three diseased and one healthy).

**Figure 3:** Comparison of four different pooling techniques (red rectangle indicates the example discussed in Section 3.2).

**Figure 4:** Schematic of proposed NCSPM.

**Figure 5:** Illustration of PatchShuffle on a grayscale COVID-19 image.

**Figure 6:** Illustration of PatchShuffle on a colorful house image.

**Figure 7:** Build PSSPNN from SPNN.

**Figure 8:** The proposed 16-way improved data augmentation method.

**Figure 9:** Proposed 16-way data augmentation results.

**Figure 10:** 3D bar plot of SPNN against other network models.

**Figure 11:** 3D bar chart of microaveraged F1 against patch size and probability.

**Figure 12:** Algorithm comparison in terms of MA F1.

**Figure 13:** Delineation of three diseased samples.

**Table 1:** Subjects and images of four categories.

Class index	Class name	$\bar{n}$	*N*_*P*_	*N*_*S*_
1	COVID-19	2.27	125	284
2	CAP	2.28	123	281
3	SPT	2.18	134	293
4	HC	2.20	139	306
Total		2.23	521	1164

**Table 2:** Abbreviation and full name.

Abbreviation	Full name
AP	Average pooling
CAP	Community-acquired pneumonia
CCT	Chest computed tomography
CI	Chest imaging
CXR	Chest X-ray
CUS	Chest ultrasound
DPD	Discrete probability distribution
FCL	Fully connected layer
FM	Feature map
FMS	Feature map size
HS	Hyperparameter size
L2P	l2-norm pooling
MA	Microaveraged
MAV	Majority voting
MDA	Multiple-way data augmentation
MP	Max pooling
NCSPM	n-conv stochastic pooling module
NWL	Number of weighted layers
SAPN	Salt-and-pepper noise
SC	Strided convolution
SLS	Slice level selection
SP	Stochastic pooling
SPNN	Stochastic pooling neural network
SPT	Second pulmonary tuberculosis
TCM	Test confusion matrix

**Table 3:** Structure of proposed 11-layer SPNN.

Index	Name	NWL	HS	FMS
1	Input			256 × 256 × 1
2	NCSPM-1	2	[3 × 3, 32] × 2	128 × 128 × 32
3	NCSPM-2	2	[3 × 3, 32]×2	64 × 64 × 32
4	NCSPM-3	2	[3 × 3, 64] × 2	32 × 32 × 64
5	NCSPM-4	2	[3 × 3, 64] × 2	16 × 16 × 64
6	NCSPM-5	1	[3 × 3, 128] × 1	8 × 8 × 128
7	Flatten			1 × 1 × 8192
8	FCL-1	1	140 × 8192, 140 × 1	1 × 1 × 140
9	FCL-2	1	4 × 140, 4 × 1	1 × 1 × 4
10	Softmax			1 × 1 × 4

**Table 4:** Pseudocode of proposed 16-way improved data augmentation.

Input	Raw image *v*(*i*)
Step 1	Eight geometric or photometric DA transforms were utilized on raw image *v*(*i*).
Step 2	A horizontal mirror image is generated.
Step 3	The raw image *v*(*i*), the mirrored image, the above 8-way DA results of the raw image, and the 8-way DA results of the horizontal mirrored image are combined to form a dataset *𝔻*(*i*).
Output	Enhanced dataset of raw image *𝔻*(*i*)

**Table 5:** Dataset splitting.

	Nontest (10-fold cross-validation)	Test (10 runs)	Total
COVID-19	|*V*_1_^ntest^| = 227	|*V*_1_^test^| = 57	|*V*_1_| = 284
CAP	|*V*_2_^ntest^| = 225	|*V*_2_^test^| = 56	|*V*_2_| = 281
SPT	|*V*_3_^ntest^| = 234	|*V*_3_^test^| = 59	|*V*_3_| = 293
HC	|*V*_4_^ntest^| = 245	|*V*_4_^test^| = 61	|*V*_4_| = 306

**Table 6:** Comparison of SPNN with four standard CNNs.

Model	Class	Sen	Prc	F1
SC-CNN	C1	93.51	93.35	93.43
	C2	86.79	91.87	89.26
	C3	94.41	91.01	92.68
	C4	94.59	93.37	93.97
	MA			92.40

AP-CNN	C1	92.86	93.02	92.94
	C2	95.76	92.93	94.32
	C3	94.26	93.95	94.11
	C4	93.22	93.22	93.22
	MA			93.18

SPNN (ours)	C1	98.07	94.59	96.30
	C2	91.79	95.19	93.45
	C3	94.92	94.92	94.92
	C4	95.25	95.40	95.32
	MA			95.02

L2P-CNN	C1	88.77	93.36	91.01
	C2	93.21	93.72	93.46
	C3	94.41	92.68	93.53
	C4	93.61	90.63	92.10
	MA			92.53

MP-CNN	C1	95.44	94.77	95.10
	C2	94.64	91.70	93.15
	C3	94.07	93.43	93.75
	C4	91.64	95.72	93.63
	MA			93.91

**Table 7:** Hyperparameter optimization of PSSPNN in terms of microaveraged F1 score.

*ε*	Patch size			
	1 × 2	2 × 2	2 × 4	3 × 3
0.01	95.19	95.54	95.15	94.98
0.05	95.49	95.79	95.45	95.11
0.10	95.24	95.28	95.54	95.41
0.15	95.24	95.11	95.28	95.06
0.20	95.06	95.15	94.85	94.72

**Table 8:** Comparison of SPNN against PSSPNN.

Model	Class	Sen	Prc	F1
SPNN (ours)	C1	98.07	94.59	96.30
	C2	91.79	95.19	93.45
	C3	94.92	94.92	94.92
	C4	95.25	95.40	95.32
	MA			95.02

PSSPN (ours)	C1	97.89	95.06	96.46
	C2	92.86	96.30	94.55
	C3	95.76	95.44	95.60
	C4	96.56	96.40	96.48
	MA			95.79

**Table 9:** Comparison with state-of-the-art approaches.

Model	Class	Sen	Prc	F1
RCBO [7]	C1	71.93	84.19	77.58
	C2	72.86	72.73	72.79
	C3	73.56	76.41	74.96
	C4	80.66	68.91	74.32
	MA			74.85

RN-50 [9]	C1	87.72	85.03	86.36
	C2	87.68	91.26	89.44
	C3	93.39	89.89	91.60
	C4	84.92	87.65	86.26
	MA			88.41

CSSNet [11]	C1	94.04	92.25	93.14
	C2	93.75	95.11	94.42
	C3	91.36	93.58	92.45
	C4	94.43	92.75	93.58
	MA			93.39

DeCovNet [13]	C1	91.05	90.58	90.81
	C2	93.75	90.99	92.35
	C3	90.51	86.97	88.70
	C4	88.69	95.58	92.01
	MA			90.94

FCONet [15]	C1	92.28	95.64	93.93
	C2	96.79	94.43	95.59
	C3	94.75	95.88	95.31
	C4	94.92	92.94	93.92
	MA			94.68

6L-CNN [8]	C1	72.46	83.94	77.78
	C2	78.93	77.82	78.37
	C3	81.86	75.00	78.28
	C4	89.84	87.54	88.67
	MA			80.94

RN-18 [10]	C1	82.81	82.66	82.73
	C2	81.07	74.43	77.61
	C3	74.24	76.98	75.58
	C4	82.13	86.38	84.20
	MA			80.04

COVNet [12]	C1	89.82	86.63	88.20
	C2	89.82	92.63	91.21
	C3	93.73	90.66	92.17
	C4	87.38	90.96	89.13
	MA			90.17

7L-CCD [14]	C1	89.47	93.58	91.48
	C2	93.93	92.44	93.18
	C3	93.73	95.18	94.45
	C4	95.08	91.34	93.17
	MA			93.09

PSSPNN (ours)	C1	97.89	95.06	96.46
	C2	92.86	96.30	94.55
	C3	95.76	95.44	95.60
	C4	96.56	96.40	96.48
	MA			95.79

## Data Availability

The data used to support the findings of this study are available from the corresponding author upon request.

## References

[1] Szigiato A. A., Anderson M., Mabon M., Germain M., Durr G. M., Labbe A. C. (2020). Usefulness of prestorage corneal swab culture in the prevention of contaminated corneal tissue in corneal transplantation. *Cornea*.

[2] Mögling R., Meijer A., Berginc N. (2020). Delayed laboratory response to covid-19 caused by molecular diagnostic contamination. *Emerging Infectious Diseases*.

[3] Ai T., Yang Z., Hou H. (2020). Correlation of chest CT and RT-PCR testing for coronavirus disease 2019 (COVID-19) in China: a report of 1014 cases. *Radiology*.

[4] Jain R., Gupta M., Taneja S., Hemanth D. J. (2021). Deep learning based detection and analysis of COVID-19 on chest X-ray images. *Applied Intelligence*.

[5] Conway H., Lau G., Zochios V. (2020). Personalizing invasive mechanical ventilation strategies in coronavirus disease 2019 (COVID-19)-associated lung injury: the utility of lung ultrasound. *Journal of Cardiothoracic and Vascular Anesthesia*.

[6] Goel A. K., DiLella D., Dotsikas G., Hilts M., Kwan D., Paxton L. (2019). Unlocking radiology reporting data: an implementation of synoptic radiology reporting in low-dose CT cancer screening. *Journal of Digital Imaging*.

[7] Wang S., Li P., Chen P. (2017). Pathological brain detection via wavelet packet Tsallis entropy and real-coded biogeography-based optimization. *Fundamenta Informaticae*.

[8] Jiang X., Zhang Y. D. (2019). Chinese sign language fingerspelling via six-layer convolutional neural network with leaky rectified linear units for therapy and rehabilitation. *Journal of Medical Imaging and Health Informatics*.

[9] Fulton L. V., Dolezel D., Harrop J., Yan Y., Fulton C. P. (2019). Classification of Alzheimer’s disease with and without imagery using gradient boosted machines and ResNet-50. *Brain Sciences*.

[10] Guo M. H., Du Y. Z. Classification of thyroid ultrasound standard plane images using ResNet-18 networks.

[11] Cohen J. P., Dao L., Roth K. (2020). Predicting COVID-19 pneumonia severity on chest X-ray with deep learning. *Cureus*.

[12] Li L., Qin L., Xu Z. (2020). Using artificial intelligence to detect COVID-19 and community-acquired pneumonia based on pulmonary CT: evaluation of the diagnostic accuracy. *Radiology*.

[13] Wang X. G., Deng X. B., Fu Q. (2020). A weakly-supervised framework for COVID-19 classification and lesion localization from chest CT. *IEEE Transactions on Medical Imaging*.

[14] Zhang Y. D., Satapathy S. C., Zhu L. Y., Gorriz J. M., Wang S. H. (2020). A seven-layer convolutional neural network for chest CT based COVID-19 diagnosis using stochastic pooling. *IEEE Sensors Journal*.

[15] Ko H., Chung H., Kang W. S. (2020). COVID-19 pneumonia diagnosis using a simple 2D deep learning framework with a single chest CT image: model development and validation. *Journal of Medical Internet Research*.

[16] Wang S.-H., Nayak D. R., Guttery D. S., Zhang X., Zhang Y. D. (2021). COVID-19 classification by CCSHNet with deep fusion using transfer learning and discriminant correlation analysis. *Information Fusion*.

[17] Zeiler M. D., Fergus R. Stochastic pooling for regularization of deep convolutional neural networks. https://arxiv.org/abs/1301.3557.

[18] Zhang Y.-D., Nayak D. R., Zhang X., Wang S.-H. (2020). Diagnosis of secondary pulmonary tuberculosis by an eight-layer improved convolutional neural network with stochastic pooling and hyperparameter optimization. *Journal of Ambient Intelligence and Humanized Computing*.

[19] Jiang X. W., Lu M., Wang S. H. (2020). An eight-layer convolutional neural network with stochastic pooling, batch normalization and dropout for fingerspelling recognition of Chinese sign language. *Multimedia Tools and Applications*.

[20] Jahanbakhshi A., Momeny M., Mahmoudi M., Zhang Y. D. (2020). Classification of sour lemons based on apparent defects using stochastic pooling mechanism in deep convolutional neural networks. *Scientia Horticulturae*.

[21] Zhou B. C., Wang X. L., Qi Q. Q. (2018). Optimal weights decoding of M-ary suprathreshold stochastic resonance in stochastic pooling network. *Chinese Journal of Physics*.

[22] Vu H., Kim H. C., Jung M., Lee J. H. (2020). fMRI volume classification using a 3D convolutional neural network robust to shifted and scaled neuronal activations. *Neuroimage*.

[23] Yang J., Ji Z. X., Niu S. J., Chen Q., Yuan S. T., Fan W. (2020). RMPPNet: residual multiple pyramid pooling network for subretinal fluid segmentation in SD-OCT images. *OSA Continuum*.

[24] Brzycki B., Siemion A. P., Croft S. (2020). Narrow-band signal localization for SETI on noisy synthetic spectrogram data. *Publications of the Astronomical Society of the Pacific*.

[25] Simonyan K., Zisserman A. Very deep convolutional networks for large-scale image recognition.

[26] Hazra A., Choudhary P., Inunganbi S., Adhikari M. (2020). Bangla-Meitei Mayek scripts handwritten character recognition using convolutional neural network. *Applied Intelligence*.

[27] Sabry Y. H., Hasan W. Z. W., Sabry A. H., Kadir M. Z. A. A., Radzi M. A. M., Shafie S. (2018). Measurement-based modeling of a semitransparent CdTe thin-film PV module based on a custom neural network. *IEEE Access*.

[28] Kang G., Dong X., Zheng L., Yang Y. Patchshuffle regularization. https://arxiv.org/abs/1707.07103.

[29] Shorten C., Khoshgoftaar T. M. (2019). A survey on image data augmentation for deep learning. *Journal of Big Data*.

[30] Wang S.-H., Govindaraj V. V., Górriz J. M., Zhang X., Zhang Y. D. (2021). Covid-19 classification by FGCNet with deep feature fusion from graph convolutional network and convolutional neural network. *Information Fusion*.

[31] Li X., Chai Y., Chen W., Ao F. Identification of early esophageal cancer based on data augmentation.

[32] Selvaraju R. R., Cogswell M., Das A., Vedantam R., Parikh D., Batra D. (2020). Grad-CAM: visual explanations from deep networks via gradient-based localization. *International Journal of Computer Vision*.

[33] Kim J., Kim J. M. (2020). Bearing fault diagnosis using Grad-CAM and acoustic emission signals. *Applied Sciences*.

[34] Akilan T., Wu Q. M. J. (2020). sEnDec: an improved image to image CNN for foreground localization. *IEEE Transactions on Intelligent Transportation Systems*.

[35] Guiga L., Roscoe A. W. Neural network security: hiding CNN parameters with guided Grad-CAM.

[36] Hossain M. S., Muhammad G., Guizani N. (2020). Explainable AI and mass surveillance system-based healthcare framework to combat COVID-I9 like pandemics. *IEEE Network*.

[37] Tosun A. B., Pullara F., Becich M. J., Taylor D. L., Fine J. L., Chennubhotla S. C. (2020). Explainable AI (xAI) for anatomic pathology. *Advances in Anatomic Pathology*.

[38] Hossain M. S. (2017). Cloud-supported cyber-physical localization framework for patients monitoring. *IEEE Systems Journal*.

[39] Hossain M. S., Muhammad G. (2018). Emotion-aware connected healthcare big data towards 5G. *IEEE Internet of Things Journal*.

[40] Liu S., Liu D. Y., Srivastava G., Połap D., Woźniak M. (2020). Overview and methods of correlation filter algorithms in object tracking. *Complex & Intelligent Systems*.

[41] Liu S., Bai W. L., Srivastava G., Machado J. A. T. (2020). Property of self-similarity between baseband and modulated signals. *Mobile Networks and Applications*.

[42] Liu S., Liu X. Y., Wang S., Muhammad K. (2021). Fuzzy-aided solution for out-of-view challenge in visual tracking under IoT-assisted complex environment. *Neural Computing & Applications*.

[43] Liu S., Wang S., Liu X., Lin C., Lv Z. (2020). Fuzzy detection aided real-time and robust visual tracking under complex environments. *IEEE Transactions on Fuzzy Systems*.

[44] Liu S., Guo C. L., al-Turjman F., Muhammad K., de Albuquerque V. H. C. (2020). Reliability of response region: a novel mechanism in visual tracking by edge computing for IIoT environments. *Mechanical Systems and Signal Processing*.

[45] Mao X., Ding L., Zhang Y., Zhan R., Li S. (2019). Knowledge-aided 2-D autofocus for spotlight SAR filtered backprojection imagery. *IEEE Transactions on Geoscience and Remote Sensing*.

[46] Mao X. H., He X. L., Li D. Q. (2018). Knowledge-aided 2-D autofocus for spotlight SAR range migration algorithm imagery. *IEEE Transactions on Geoscience and Remote Sensing*.

[47] Mao X. H., Zhu D. Y. (2016). Two-dimensional autofocus for spotlight SAR polar format imagery. *IEEE Transactions on Computational Imaging*.

[48] Xia K., Zhang Y., Jiang Y. (2020). TSK fuzzy system for multi-view data discovery underlying label relaxation and cross-rule & cross-view sparsity regularizations. *IEEE Transactions on Industrial Informatics*.

[49] Xia K., Gu X., Chen B. (2020). Cross-dataset transfer driver expression recognition via global discriminative and local structure knowledge exploitation in shared projection subspace. *IEEE Transactions on Intelligent Transportation Systems*.

[50] Xia K., Ni T., Yin H., Chen B. (2020). Cross-domain classification model with knowledge utilization maximization for recognition of epileptic EEG signals. *IEEE/ACM Transactions on Computational Biology and Bioinformatics*.

